The article "Artificial Intelligence Algorithm-Based Differential Diagnosis of Crohn's Disease and Ulcerative Colitis by CT Image" was retracted in 2023. Reasons: signs of a paper mill; compromised peer review; unreliable results or conclusions.

# Artificial Intelligence Algorithm-Based Differential Diagnosis of Crohn's Disease and Ulcerative Colitis by CT Image

**DOI:** 10.1155/2022/3871994

**Published:** 2022-04-04

**Authors:** Fangyun Jiang, Xiaoping Fu, Kai Kuang, Dan Fan

**Affiliations:** ^1^Department of Gastroenterology, The Third Affiliated Hospital, Hengyang Medical School, University of South China, Hengyang, Hunan 421001, China; ^2^Department of Neurosurgery, The Third Affiliated Hospital, Hengyang Medical School, University of South China, Hengyang, Hunan 421001, China

## Abstract

The aim of this study was to investigate the effect of low-dose CT enterography (CTE) based on modified guided image filtering (GIF) algorithm in the differential diagnosis of ulcerative colitis (UC) and Crohn's disease (CD). *Methods*. One hundred and twenty patients with suspected diagnosis of IBD were studied. They were randomly divided into control group (routine CT examination) and observation group (low-dose CTE examination based on improved GIF algorithm), with 60 cases in each group. Comprehensive diagnosis was used as the standard to assess the diagnostic effect. *Results*. (1) The peak signal-to-noise ratio (PSNR) (26.02 dB) and structural similarity (SSIM) (0.8921) of the algorithm were higher than those of GIF (17.22 dB/0.8491), weighted guided image filtering (WGIF) (23.78 dB/0.8489), and gradient domain guided image filtering (GGIF) (23.77 dB/0.7567) (*P* < 0.05); (2) the diagnostic sensitivity (91.49%), specificity (92.31%), accuracy (91.67%), positive predictive value (97.73%), and negative predictive value (75%) of the observation group were higher than those of the control group (*P* < 0.05); the sensitivity and specificity of CTE in the diagnosis of UD and CD were 96.77% and 81.25% and 98.33% and 93.33%, respectively (*P* < 0.05); there were significant differences in symmetrical intestinal wall thickening and smooth serosal surface between UD and CD (*P* < 0.05). *Conclusion*. (1) The improved GIF algorithm has a more effective application value in the denoising processing of low-dose CT images and can better improve the image quality; (2) the accuracy of CTE in the diagnosis of IBD is high, and CTE is of great value in the differential diagnosis of UD and CD.

## 1. Introduction

Inflammatory bowel disease (IBD) is a chronic nonspecific intestinal inflammatory disease [1, 2], which has a high incidence in Western countries, and with the development of society, the probability of IBD disease in China has gradually increased [3]. Ulcerative colitis (UC) and Crohn's disease (CD) are two subtypes of IBD [4, 5]. UC is relatively common in clinical practice, and the main sites of disease are in the sigmoid colon and rectum, and clinical studies suggest that the main factors in the pathogenesis of UC are infection, immunity, genetics, spirit, and environment [6]. While the pathogenesis of CD is more complex, it is not yet clarified in clinical practice, and the site of CD pathogenesis is relatively wide and may involve the entire intestine [7]. However, practice showed that there is some difficulty in the differential diagnosis between UC and CD diseases in clinical practice. The clinical manifestations of UC and CD are not significantly specific, and all of them are dominated by abdominal pain, weight loss, and watery or viscous purulent bloody stools [8].

The article "Artificial Intelligence Algorithm-Based Differential Diagnosis of Crohn's Disease and Ulcerative Colitis by CT Image" was retracted in 2023. Reasons: signs of a paper mill; compromised peer review; unreliable results or conclusions.

The main methods used for the diagnosis of IBD diseases in clinical practice are colonoscopy biopsy, endoscopic ultrasonography, CT, and MRI. Among them, colonoscopy biopsy is invasive although it is the gold standard [9]. Endoscopic ultrasonography only reflects anatomical morphological changes and has a greater dependence on operator experience [10]. CT and MRI examinations reduce the accuracy of diagnosis due to the interference of some uncertain factors in the nature of the intestine, such as protracted tortuosity of the intestine, peristalsis leading to changes in the location and shape of the intestine [11]. Thus, CT enterography (CTE) technology is developed. CTE is the uniform dilatation of the small intestine by oral contrast medium, and images are obtained by continuous scanning using CT after intravenous enhancement [12]. Studies showed that CTE has more advantages in displaying intestinal wall, intraluminal lesions, with high temporal and spatial resolution, and can also observe the small intestine from multiple planes [13]. However, there are few studies on CTE for IBD disease diagnosis. Therefore, in this study, CTE will be used to study the differential diagnosis between UC and CD.

Studies found that due to the high radiation of CT scan, it will bring some adverse reactions to patients and even have the risk of carcinogenesis [14]. Thus, low-dose CT received much attention; however, with the reduction of radiation dose, the quality of CT images will also be reduced. Therefore, removing the noise of low-dose CT images is the hot spot to researchers [15]. With the development of artificial intelligence algorithms in recent years, many applied studies were obtained in the field of imaging, and most of them have achieved good results [16, 17]. Guided image filtering (GIF) is a representative local algorithm in recent years, and its calculation method is also simple [18]. However, due to its fixed regularization coefficient, the image will produce halo, including weighted guided image filtering (WGIF) and gradient domain guided image filtering (GGIF) [19, 20]. Therefore, it is proposed to improve the GIF algorithm and add an edge-aware weighting factor to the regularization coefficient to solve the above problems [21], and good results are obtained.

The article "Artificial Intelligence Algorithm-Based Differential Diagnosis of Crohn's Disease and Ulcerative Colitis by CT Image" was retracted in 2023. Reasons: signs of a paper mill; compromised peer review; unreliable results or conclusions.

In summary, in order to provide more and more effective research basis for clinical differential diagnosis and treatment of IBD diseases, low-dose CTE based on improved GIF algorithm will be used to examine and diagnose UD and CD patients, evaluate the differential diagnosis effect of CTE in UD and CD, and observe the specific performance of UD and CD in CTE images.

## 2. Research Methods

### 2.1. Objects

In this study, 120 patients with suspected IBD admitted to hospital from June 2018 to May 2021 were randomly selected as the study subjects. Among them, there were 71 male patients and 49 female patients, aged between 20 and 50 years, with an average age of 34.78 ± 12.45 years. There were 72 patients with clinical manifestations of abdominal pain, 103 patients with diarrhea, 56 patients with tenesmus, 49 patients with viscous purulent bloody stools, and 44 patients with fever. A total of 120 patients were randomly divided into two groups. The control group was examined and diagnosed by conventional CT images. The observation group was examined and diagnosed by low-dose CTE images based on the improved GIF algorithm, with 60 patients in each group. The results of imaging diagnosis and comprehensive diagnosis (clinical manifestations, imaging examination, endoscopy, and colonoscopy biopsy) were compared between the two groups to evaluate the diagnostic effect. The CTE features of the patients were observed in the observation group, and the CTE features between UC and CD were compared. This study had been approved by the medical ethics committee of the hospital. All the patients and their families understood the study and signed informed consent.

Inclusion criteria: patients over 18 years of age; all patients were diagnosed with IBD diagnostic criteria [22]; patients had informed consent and agreed to this study; patients with complete clinical data.

Exclusion criteria: patients with severe organ dysfunction and malignant tumors; patients with ischemic, infectious, postradiotherapy, and other intestinal diseases; pregnant or lactating women; excluding patients with anisodamine contraindications and acute intestinal obstruction.

### 2.2. CTE Examination

128-slice spiral CT was used for scanning examinations. Patients were required to fast for more than 8 hours before examination. 2,000 mL of 2.5% mannitol infiltration solution was orally administered within 1 hour before scanning, once every 15 minutes, divided into 4 doses of 500 mL each time. 10 mg anisodamine was intravenously injected 10 minutes before the scan to inhibit intestinal peristalsis (the dose was adjusted according to the patient's individual condition). Scan range: top of diaphragm–superior border of pubic symphysis. Scanning mode: plain scan, enhanced arterial phase, and venous phase. Scanning parameters: matrix—512 × 512, field of view—350 mm, tube voltage—120 kV, and tube current—300~350 mA. Contrast-enhanced scanning: 100 mL of Ultravist with a concentration of 370 mgI·mL^−1^ was intravenously injected through the antecubital vein with a high-pressure syringe at an injection rate of 3~4 mL·s^−1^. Afterwards, arterial phase scanning was performed using an automatic tracing technique (CT threshold was set at 120 Hu), and venous phase scanning was performed with a delay of 30 s after the end.

The article "Artificial Intelligence Algorithm-Based Differential Diagnosis of Crohn's Disease and Ulcerative Colitis by CT Image" was retracted in 2023. Reasons: signs of a paper mill; compromised peer review; unreliable results or conclusions.

### 2.3. Low-Dose CT Based on Improved GIF Algorithm

#### 2.3.1. GIF Algorithm

In the GIF algorithm, the linear relationship between the output image *Q* and the guided image *I* is as follows.

(1) $$\begin{array}{c} Q_{i}=a_{k}I_{i}+b_{k},\;\forall i\in \omega_{k}. \end{array}$$

In the above equation, *i* refers to the spatial coordinates of pixels in the output image *Q*, (*a*_*k*_, *b*_*k*_) refers to the linear coefficient, and (*a*_*k*_, *b*_*k*_) is a constant in the window *ω*_*k*_ when the pixel is *I*_*i*_.

GIF algorithm has good characteristics in edge preserving, mainly because of the same gradient of *Q* and *I*, namely, ∇*Q* = *a*∇*I*. Therefore, GIF is widely used. The objective function is defined as follows.

(2) $$\begin{array}{c} E\left(a_{k},b_{k}\right)=\min\underset{i\in \omega_{k}}{\sum }\left(\left(a_{k}I_{i}+b_{k}-p_{i}\right)+\lambda a_{k}^{2}\right). \end{array}$$

*p* refers to the input image, and *λ* refers to the regularization coefficient. This equation has two functions: first, it reduces the difference between *Q* and *p*; second: it avoids *a*_*k*_ be too large. By solving the above equation, the following equations can be obtained.

(3) $$\begin{array}{c} a_{k}=\frac{\left(1/\left|\omega \right|\right)\sum_{i\in \omega_{k}}I_{i}p_{i}-\mu_{k}{\bar{p}}_{k}}{\sigma_{k}^{2}+\lambda },\\ b_{k}={\bar{p}}_{k}-a_{k}\mu_{k}. \end{array}$$

The above *μ*_*k*_ and *σ*_*k*_^2^ separately represent the mean and variance of the guided image *I* in the window *ω*_*k*_. |*ω*| represents the total pixel in the window *ω*_*k*_, and ${\bar{p}}_{k}$ represents the mean value of the input image *p* in the window *ω*_*k*_.

In the GIF algorithm, the edge weight factor will change with the spatial position of the image. Therefore, to a certain extent, it can avoid or weaken the halo and guide each pixel *I*_*i*′_ in the image. The following edge weight factor is defined.

(4) $$\begin{array}{c} \Gamma_{K}\left(I_{i\prime }\right)=\frac{1}{N}\overset{N}{\underset{i=1}{\sum }}\frac{\sigma_{K,1}^{2}\left(I_{i\prime }\right)}{\sigma_{K,1}^{2}\left(I_{i}\right)}. \end{array}$$

*N* represents the number of pixels in an image and *σ*_*K*,1_^2^(*I*_*i*′_)*N* represents the variance of pixels *I*_*i*′_ in the window *ω*_*K*,1_.

The article "Artificial Intelligence Algorithm-Based Differential Diagnosis of Crohn's Disease and Ulcerative Colitis by CT Image" was retracted in 2023. Reasons: signs of a paper mill; compromised peer review; unreliable results or conclusions.

#### 2.3.2. Improved GIF Algorithm

As shown in Equation (4), if the equation is used for calculation, it may lead to a large deviation between the final calculation results and the actual results, which will misjudge the properties of pixels in the window. Therefore, some people improved the calculation of the edge weight factor, which is expressed as follows.

(5) $$\begin{array}{c} \Gamma_{K}\left(I_{i\prime }\right)=\frac{1}{\left|\Omega_{K,\xi_{1}}\right|}\underset{i=K,\xi_{1}}{\sum }\frac{\sigma_{K,\xi_{1}}^{2}\left(I_{i\prime }\right)}{\sigma_{K,\xi_{1}}^{2}\left(I_{i}\right)}. \end{array}$$

|*Ω*_*K*,*ξ*_1__| represents the number of pixels in the window *Ω*_*K*,*ξ*_1__. In this equation, the ratio of each pixel variance to the pixel variance in the filter window is taken as the measurement standard so that the whole image is reduced to a local window, thereby improving the accuracy.

It is supposed that the detail layer image is *r*, and the base layer image is *Q*. Then, its expression can be expressed as follows.

(6) $$\begin{array}{c} r=I-Q. \end{array}$$

The image *r*′ obtained by enhancing the detail layer can be expressed as follows.

(7) $$\begin{array}{c} r^{\prime }=\alpha \cdot r,\\ r^{\prime }=\alpha \cdot \left(I-Q\right). \end{array}$$

*α* represents detail layer gain. Then, the output image *f* can be expressed as follows.

(8) $$\begin{array}{c} f=Q+r^{\prime }. \end{array}$$

By substituting Equation (1), the following equation can be obtained.

(9) $$\begin{array}{c} r^{\prime }=\alpha \cdot \left(I-aI-b\right). \end{array}$$

It also can be represented as

(10) $$\begin{array}{c} r^{\prime }=\alpha \cdot \left(1-a\right)I-\alpha \cdot b. \end{array}$$

According to Equation (10), the gradient of the detail layer can be calculated as follows.

(11) $$\begin{array}{c} \nabla r^{\prime }=\alpha \cdot \left(1-a\right)\nabla I. \end{array}$$

According to Equation (1), the gradient of the base layer can be calculated as follows.

(12) $$\begin{array}{c} \nabla Q=a\cdot \nabla I. \end{array}$$

Since the enhanced detail layer gradient may not be greater than the base layer, the following definition is required.

(13) $$\begin{array}{c} \nabla r^{}\nabla Q. \end{array}$$

Combining Equation (11) with Equation (12), the following expressions can be obtained.

(14) $$\begin{array}{c} \alpha \cdot \left(1-a\right)\nabla I\leq a\cdot \nabla I,\\ \alpha \leq \frac{a}{1-a}. \end{array}$$

The article "Artificial Intelligence Algorithm-Based Differential Diagnosis of Crohn's Disease and Ulcerative Colitis by CT Image" was retracted in 2023. Reasons: signs of a paper mill; compromised peer review; unreliable results or conclusions.

#### 2.3.3. Evaluation Indicators

In order to quantitatively evaluate the image quality, two commonly used indicators are given: peak signal-to-noise ratio (PSNR) and structural similarity (SSIM). PSNR measures the denoising ability, and the higher the results, the better the denoising effect. SSIM is based on structural similarity, to evaluate the quality of the image, the value between -1 and 1, the greater the value, the better the image quality. The specific expression is as follows.

(15) $$\begin{array}{c} \text{PSNR}=10\log_{10}\left(\frac{M}{{\left\|\bar{I}-I\right\|}_{2}^{2}}\right). \end{array}$$

*I* represents the noiseless CT image, $\bar{I}$ represents the denoised image, and *M* represents the number of pixels in the image.

(16) $$\begin{array}{c} \text{SSIM}\left(x,\text{y}\right)=\frac{\left(2\alpha_{x}\alpha_{y}+e_{1}\right)\left(2\beta_{xy}+e_{2}\right)}{\left(\alpha_{x}^{2}+\alpha_{y}^{2}+e_{1}\right)\left(\beta_{x}^{2}+\beta_{y}^{2}+e_{2}\right)}. \end{array}$$

*α*_*x*_ is the average value of *x*; *α*_*y*_ is the average value of *y*; *β*_*x*_^2^ is the variance of *x*; *β*_*y*_^2^ is variance of *y*; *β*_*xy*_ is the covariance of *x* and *y*.

### 2.4. Observation Indexes

1. The imaging findings and diagnostic results of UC and CD in the two groups of examination methods were evaluated, and the sensitivity, specificity, accuracy, negative predictive value, and positive predictive value were calculated. The specific calculation methods are as follows:

(17) $$\begin{array}{c} \text{Sensitivity}=\frac{A}{A+B+C+D}\times 100\%,\\ \text{Specificity}=\frac{D}{A+B+C+D}\times 100\%,\\ \text{Accuracy}=\frac{A+D}{A+B+C+D}\times 100\%,\\ \text{Negative predictive value}=\frac{D}{C+D}\times 100\%,\\ \text{Positive predictive value}=\frac{A}{A+B}\times 100\%. \end{array}$$

*A* represents the number of samples with true positive results, *B* represents the number of samples with false positive results, *C* represents the number of samples with false negative results, and *D* represents the number of samples with true negative results.

(2) The intestinal lesions of UC and CD diseases under CTE in the observation group, including wall lesions, mode and location of lesion involvement, intestinal morphology, and extraintestinal manifestations, were compared

### 2.5. Statistical Methods

SPSS 22.0 statistical software was used to analyze the data. The measurement data conforming to normal distribution were expressed as mean ± standard deviation ($\overset{¯}{x}\pm s$), with two decimal places reserved. The paired *t-*test was used for comparison within two groups, and the independent sample *t-*test was used for comparison between two groups. The quantitative data conforming to skewed distribution were expressed as median (range), and the Wilcoxon rank sum test was used for comparison between two groups. Enumeration data were expressed as percentages (%) to one decimal place, and the *χ*^2^ test or continuity correction of *χ*^2^ test was used for comparison between two groups. *P* values were rounded to three decimal places, and *P* < 0.05 was considered statistically significant.

The article "Artificial Intelligence Algorithm-Based Differential Diagnosis of Crohn's Disease and Ulcerative Colitis by CT Image" was retracted in 2023. Reasons: signs of a paper mill; compromised peer review; unreliable results or conclusions.

## 3. Results

### 3.1. Application Effect of Improved GIF Algorithm

The image processing effect of this algorithm with GIF, WGIF, and GGIF algorithms was compared for low-dose CT (Figure 1). The detailed results in the yellow box showed that although GIF, WGIF, and GGIF algorithms can enhance the details of the image, the noise was also amplified, while the algorithm in this study not only enhanced the details of the image but also effectively inhibited the noise of the image and enhanced the medical characteristics.

### 3.2. Comparison of Denoising Effect

Figure 2 shows the comparison of PSNR and SSIM between the proposed algorithm and GIF, WGIF, and GGIF algorithms for low-dose CT image processing. The results show that the PSNR and SSIM values of the proposed algorithm are higher than those of the other three algorithms (*P* < 0.05).

### 3.3. Comparison of General Data

The general clinical data of the two groups of patients were compared. In the control group, the number of males was 34 (51.52%) and the number of females was 27 (48.21%); in the observation group, the number of males was 32 (48.48%) and the number of females was 29 (51.79%). The mean age was 33.98 ± 12.88 years in the control group and 35.11 ± 11.57 years in the observation group. The distribution of clinical manifestations is illustrated in Figure 3. After analysis and comparison, the difference in the distribution of general clinical data between the two groups had no statistical significance (*P* > 0.05), suggesting the feasibility of comparison in this study.

### 3.4. Comparison of Diagnostic Effect

Table 1 shows the statistics of the conventional CT examination and comprehensive diagnosis results of IBD patients in the control group, and Table 2 shows the CTE examination and comprehensive diagnosis results of IBD patients in the observation group based on the improved GIF algorithm. After calculation, in 42 cases of IBD patients in the control group, the diagnostic sensitivity was 69.05%, specificity was 44.44%, accuracy was 61.67%, positive predictive value was 74.36%, and negative predictive value was 38.10%. There were 47 cases of IBD patients in the observation group; the diagnostic sensitivity was 91.49%, specificity was 92.31%, accuracy was 91.67%, positive predictive value was 97.73%, and negative predictive value was 75%.

The article "Artificial Intelligence Algorithm-Based Differential Diagnosis of Crohn's Disease and Ulcerative Colitis by CT Image" was retracted in 2023. Reasons: signs of a paper mill; compromised peer review; unreliable results or conclusions.

### 3.5. Comparison of Diagnostic Effects of UC and CD in the Observation Group

The diagnostic effect of CTE based on improved GIF algorithm on UC and CD was analyzed. The results are shown in Tables 3 and 4. The results showed that the diagnostic sensitivity, specificity, accuracy, positive predictive value, and negative predictive value of CTE based on the improved GIF algorithm for UC were 96.77%, 100%, 98.33%, 100%, and 96.67%, respectively. The diagnostic sensitivity of CD was 81.25%, the specificity was 97.73%, the accuracy was 93.33%, the positive predictive value was 92.86%, and the negative predictive value was 93.48%.

### 3.6. CTE Image Features of UC and CD

#### 3.6.1. Characteristics of Intestinal Wall Lesions

Figure 4 is the statistical characteristics of intestinal wall lesions in CTE images of UC and CD diseases. The results show that in 30 patients with UC, 30 cases had intestinal wall thickening (>4 mm) (100%), 29 cases had thickening symmetry (96.67%), 29 cases had abnormal enhancement (96.67%), and 29 cases had smooth serosa surface (96.67%). In 13 patients with CD, 11 cases (84.61%) had intestinal wall thickening (>4 mm), 1 case (7.69%) had symmetrical thickening, 12 cases (92.31%) had abnormal enhancement, and 2 cases (15.38%) had smooth serosa surface. After comparison, there was no significant abnormality in the probability of thickening and abnormal enhancement of intestinal wall between UC and CD (*P* > 0.05), while the proportion of cases with symmetric thickening and smooth serosa surface was significantly different (*P* < 0.05).  Figure 5 shows the specific CTE manifestations.

#### 3.6.2. Mode and Location of Lesions Involved

Figure 6 shows the results of CTE images of UC and CD diseases on the lesion involvement mode and location. The results showed that in 30 patients with UC, there were 2 cases of stage involvement (6.67%), 28 cases of continuity (93.33%), 0 cases of jejunum disease location (0%), 0 cases of ileum/cecum (0%), and 29 cases of rectum and colon (96.67%). Among the 13 CD patients, there were 12 cases of stage involvement (92.31%), 1 case of continuity (7.69%), 7 cases of jejunum disease location (53.85%), 12 cases (92.31%) in ileum/cecum, and 7 cases (53.85%) in rectum and colon.

#### 3.6.3. Intestinal Morphology and Extraintestinal Manifestations

Figure 7 shows the examination results of CTE images on intestinal morphology in patients with UC and CD diseases. The results showed that in 30 patients with UC, 24 patients (80%) had colon bag disappearance and intestinal stiffness, and in 13 patients with CD, 3 patients (23.08%) had colon bag disappearance and intestinal stiffness. Compared with the results of extraintestinal manifestations, the mesenteric density increased in 18 cases (60%), lymph node enlargement in 19 cases (63.33%), comb sign in 12 cases (40%), cellulitis in 2 cases (6.67%), complicated with abdominal/perianal abscess, fistula in 2 cases (6.67%), and complicated with intestinal obstruction in 2 cases (6.67%). Among 13 CD patients, mesenteric density increased in 8 cases (61.54%), lymph node enlargement in 8 cases (61.54%), comb sign in 5 cases (38.46%), cellulitis in 7 cases (53.85%), complicated with abdominal/perianal abscess, fistula in 6 cases (46.15%), and complicated with intestinal obstruction in 6 cases (46.15%).

The article "Artificial Intelligence Algorithm-Based Differential Diagnosis of Crohn's Disease and Ulcerative Colitis by CT Image" was retracted in 2023. Reasons: signs of a paper mill; compromised peer review; unreliable results or conclusions.

## 4. Discussion

With the rapid development of medical technology, there are more and more methods used for the examination of intestinal diseases in clinical practice, such as colonoscopy [23] and capsule endoscopy [24], which are widely used in clinical practice. However, the above examinations cannot examine the conditions inside and outside the intestinal canal at the same time and will bring certain complications to patients. Thus, CTE examination is proposed, and studies showed that CTE examination can perform a full range of examinations for the extent of the lesion, internal and external involvement of the bowel [25]. CTE gives the patient contrast medium and injects it based on CT examination, and the final image still needs CT scan.

UC and CD in IBD diseases have no obvious specificity due to clinical manifestations, and routine examination is also prone to missed diagnosis and misdiagnosis due to the particularity of small intestinal structure. Therefore, the differential diagnosis of UC and CD has become the focus of clinical research [26]. There are many previous studies on the application of CTE in CD, but there are relatively few studies on the differential diagnosis of CTE between UC and CD. This study investigated the use of CTE in UC and CD. In this study, the diagnostic effect of conventional CT and CTE on IBD diseases was compared. In order to reduce the radiation caused by CT scan to patients, low-dose CT was used for scanning, and the improved GIF algorithm was used to denoise the CT scan image so that it reached the degree of conventional CT image in the image display. The processing results were compared with GIF, WGIF, and GGIF algorithms. The results showed that the PSNR and SSIM of this algorithm are higher than those of GIF, WGIF, and GGIF. It is suggested that the improved GIF algorithm has more effective results in the processing of low-dose CT images, namely, it is effective to improve the edge weight coefficient and detail layer gain [27]. Li et al. [28] combined the sparse domain regularized strip decomposition (SDRSD) method with the GIF algorithm and achieved good results. He et al. [29] also improved GIF and used it on the image processing of low-dose CT, and the results were basically consistent with this study.

The article "Artificial Intelligence Algorithm-Based Differential Diagnosis of Crohn's Disease and Ulcerative Colitis by CT Image" was retracted in 2023. Reasons: signs of a paper mill; compromised peer review; unreliable results or conclusions.

The CTE images obtained by low-dose CT scanning with noise removal were used in the disease diagnosis of IBD and compared with conventional CT examination, and the diagnostic sensitivity (91.49%), specificity (92.31%), accuracy (91.67%), positive predictive value (97.73%), and negative predictive value (75%) of the observation group were higher than those of the control group (69.05%, 44.44%, 61.67%, 74.36%, and 38.10%). These results suggest that CTE is more effective in the diagnosis of IBD diseases and has clinical application value [30, 31]. The above studies suggest a good application effect of CTE in IBD diseases. It is consistent with the results of this study. Based on the above findings that CTE has more accurate diagnostic results, the diagnostic effect and imaging characteristics of CTE for UC and CD were analyzed in combination with comprehensive diagnosis. The results showed that the diagnostic efficacy of CTE for UC and CD was higher than 80%, and the sensitivity and specificity of CTE in the diagnosis of UC and CD were 96.77% and 81.25% and 98.33% and 93.33%, respectively, suggesting that the differential diagnosis effect was good. It is proposed that both UC and CD have manifestations of intestinal wall thickening, but there are some differences in the characteristics of intestinal wall thickening [32]. The statistical results of this study showed that among UC patients, 96.67% had symmetric intestinal wall thickening, and among CD patients, 7.69% had symmetric intestinal wall thickening. Therefore, UC was mainly characterized by symmetrical intestinal wall thickening, while CD was mainly characterized by asymmetric intestinal wall thickening. The proportion of patients with UC (96.67%) was significantly higher than that of CD (15.38%) in the comparison of whether the plasma membrane surface of intestinal wall was smooth. This study concluded that most patients with UC were continuous lesions (93.33%), mainly in the rectum and colon (96.67%), and CD was mostly stage full-thickness involvement of small intestinal wall (92.31%). Some studies pointed out that the probability of colon bag disappearance and intestinal stiffness in patients with UC is higher [33], which is consistent with the results of this study (UC vs. CD: 80% vs. 23.08%). Moreover, this study also found that CD lesions involving extraintestinal causes of cellulitis, abdominal/perianal abscess, fistula, and intestinal obstruction are more likely (53.85% vs. 6.67%/46.15% vs. 6.67%/46.15% vs. 6.67%).

The article "Artificial Intelligence Algorithm-Based Differential Diagnosis of Crohn's Disease and Ulcerative Colitis by CT Image" was retracted in 2023. Reasons: signs of a paper mill; compromised peer review; unreliable results or conclusions.

## 5. Conclusion

In this study, low-dose CTE based on the improved GIF algorithm was used to examine and diagnose UC and CD, and the specific manifestations of UC and CD in CTE images were observed to evaluate its application effect in the differential diagnosis of UC and CD. Based on the above results, it can be concluded that (1) the improved GIF algorithm has a more effective application value in the denoising processing of low-dose CT images and can better improve the image quality; (2) the better accuracy of CTE in the diagnosis of IBD diseases, and there are differences in the performance of CD and UC in CTE, and CTE is of great value in the differential diagnosis of the two diseases. However, in this study, only the patients in the observation group were used to analyze the CTE characteristics of UC and CD, and the small number of study samples may cause some errors in the results. However, in the general trend, CTE diagnosis has a good application prospect in the diagnosis of IBD and the differential diagnosis of UC and CD.

## Figures and Tables

**Figure 1:** Low-dose CT image processing effect comparison. The detailed image site is displayed in the yellow box: (a) low-dose CT image; (b) GIF algorithm; (c) WGIF algorithm; (d) GGIF algorithm; (e) the algorithm in this study; (f) normal dose CT.

**Figure 2:** Comparison of denoising effect. ^∗^Compared with the algorithm, *P* < 0.05.

**Figure 3:** Analysis of general data: (a) abdominal pain; (b) diarrhea; (c) tenesmus; (d) viscous purulent bloody stool; (e) fever.

**Figure 4:** Characteristic statistics of CTE images of UC and CD intestinal wall lesions: (a) intestinal wall thickening (>4 mm); (b) symmetrical thickening; (c) abnormal enhancement of intestinal wall; (d) smooth serosa surface. ^∗^Compared with UC, *P* < 0.05.

**Figure 5:** CTE images of intestinal wall lesions: (a) wall of the ascending colon of UC patient was thickened, with layered enhancement (presenting target sign), indicated by red arrow; (b) wall of the colon of UC patient was asymmetrically thickened, indicated by red arrow; (c) intestinal wall of the jejunum of CD patient was abnormally thickened and enhanced, indicated by red arrow; (d) intestinal wall of CD patient was layered enhancement, presenting target sign, indicated by red arrow.

The article "Artificial Intelligence Algorithm-Based Differential Diagnosis of Crohn's Disease and Ulcerative Colitis by CT Image" was retracted in 2023. Reasons: signs of a paper mill; compromised peer review; unreliable results or conclusions.

**Figure 6:** Statistical analyses of CTE image characteristics of involved modes and sites of UC and CD lesions. A, B, C, D, and E represent stage, continuous, jejunum, ileum/ileocecum, and rectum and colon, respectively. UC and CD represent jejunal and ileal segmental wall thickening and jejunal and ileal continuous wall thickening, respectively. ^∗^Compared with UC, *P* < 0.05.

**Figure 7:** Examination results of UC and CD extraintestinal manifestations: (a) increased mesenteric density; (b) lymph node enlargement; (c) comb sign; (d) cellulitis; (e) abdominal/perianal abscess, fistula; (f) intestinal obstruction. ^∗^Compared with UC, *P* < 0.05.

**Table 1:** Statistics of diagnosis results in the control group.

Control group (*n* = 60 cases)		Comprehensive diagnosis		Total
CT examination	IBD	29	10	39
	Non-IBD	13	8	21
Total		42	18	60

**Table 2:** Statistics of diagnosis results in the observation group.

Observation group (*n* = 60 cases)		Comprehensive diagnosis		Total
		IBD	Non-IBD	
CT examination	IBD	43	1	44
	Non-IBD	4	12	16
Total		47	13	60

**Table 3:** UC diagnostic result statistics.

		Comprehensive diagnosis (*n* = 60 cases)		Total
		UC	Non-UC	
CTE examination (*n* = 60 cases)	UC	30	0	30
	Non-UC	1	29	30
Total		31	29	60

**Table 4:** CD diagnostic result statistics.

		Comprehensive diagnosis (*n* = 60 cases)		Total
		CD	Non-CD	
CTE examination (*n* = 60 cases)	CD	13	1	14
	Non-CD	3	43	46
Total		16	44	60

## Data Availability

The data used to support the findings of this study are available from the corresponding author upon request.
